# Epidemiological Analysis and Prognosis of Conjunctival Cancer in the Past Twenty Years: A Population-Based Retrospective Study Using SEER Data

**DOI:** 10.1155/2020/1203938

**Published:** 2020-07-07

**Authors:** Yumei Diao, Xiaoqi Li, Yan Huo, Zongyuan Li, Qinghua Yang, Yifei Huang, Liqiang Wang

**Affiliations:** ^1^Department of Ophthalmology, The 1st Medical Center of Chinese PLA General Hospital, Beijing 100853, China; ^2^Department of Ophthalmology, The PLA Second Artillery General Hospital, Beijing 100088, China

## Abstract

Epidemiological studies of malignant primary conjunctival tumors are rare. We extracted data pertaining to primary site-labeled conjunctival cancer patients present within the Surveillance, Epidemiology, and End Results (SEER) database from 1992 to 2001 and from 2002 to 2011. The Kaplan-Meier approach was used for comparisons of overall survival (OS) between patients, while OS-related risk factors were identified via a Cox proportional hazards regression approach. We then constructed a nomogram that could be used to predict the 3- and 5-year OS, with the accuracy of this predictive model based on receiver operating characteristic (ROC) curve. We observed a significant reduction in age-adjusted incidence of conjunctival cancer in the 50-69-year-old age group of the 2002-2011 cohort relative to the 1992-2001 cohort (APC, *P* < 0.05). There were no significant differences in OS between the 1992-2001 and 2002-2011 conjunctival cancer patient cohorts. Being ≥30 years old (*P* < 0.05), male (*P* < 0.001), single (*P* < 0.05), divorced (*P* < 0.001), or widowed (*P* < 0.001) were all associated with an increased OS-related risk of primary conjunctival cancer (1992-2011). Our nomogram was able to accurately predict 3- and 5-year OS in conjunctival cancer patients. In verification mode, the 3-year area under the curve (AUC) was 0.697 and the 5-year AUC was 0.752. We found that age, sex, and marital status were all associated with primary conjunctival cancer survival. Our results further suggest that conjunctival cancer incidence and survival rates have been relatively stable over the last two decades, and using these data, we were able to generate a satisfactory risk prediction model for this disease.

## 1. Introduction

Conjunctival cancers can arise due to the metastasis of other cancers such as breast cancer [1], mucosal gastric cancer [2], or epidermodysplasia verruciformis [3], or they can manifest as primary cancers [4]. While conjunctival cancers are relatively uncommon, one study of 5002 cases of patients with these tumors that were referred to an ocular oncology tertiary care center found that they were malignant in up to 30% of patients (primarily in cases of melanoma, squamous cell carcinoma, and lymphoma) [5]. Among children, malignant conjunctival tumors account for over 3% of total malignancies [6].

The etiology of this disease, and particularly of primary conjunctival cancer, is still not well defined. Causes underlying its development are likely multifactorial, being influenced by age, sex, ethnicity, systemic diseases, and environmental factors [7–12]. Conjunctival cancers can cause vision loss, metastasis, and eventually death [13]. To date, few studies have explored risk factors associated with the epidemiology of primary site-labeled conjunctival tumors, patient survival duration, and patient prognosis.

As such, in the present study, we assessed a number of epidemiological trends associated with such tumor age-adjusted incidence rate trends, cause-specific survival, and associated risk factors related to survival time in cases of malignant primary conjunctival tumors diagnosed in 1992–2001 and in 2002–2011 using the SEER database. By leveraging these data, we were able to develop and validate a clinical prognostic model for patients with malignant primary site-labeled conjunctival tumors.

## 2. Methods

We obtained data pertaining to cases of conjunctival cancer for which primary site information was available within the population-based database managed by the National Cancer Institute SEER Program. Only data pertaining to primary conjunctival cancer cases with site codes corresponding to the conjunctiva (C69.0) and the cornea (C69.1) were considered in the present analysis. We elected to include cases of corneal cancer in this study as primary corneal cancer is an extremely rare disease, and in most cases, such tumors are thought to represent extensions of conjunctival cancers from the limbus.

After extracting these data, we separated patients based upon their year of diagnosis into two decade-based cohorts: 1992-2001 and 2002-2011. We then compiled basic demographic information pertaining to these 2369 patients, including age, sex, ethnicity, and marital status (Table 1). We further calculated age-adjusted incidence trends, with rates being per 100,000 persons and being age-adjusted to the 2000 US Std population standard (age-adjusted reference population). A weighted least-squares approach was used to calculate annual percent change (APC) values. For further analyses, we excluded all data for which patient age, sex, ethnicity, or marital status was undefined. We then used a Kaplan-Meier approach to compare cause-specific survival rates between patient subsets, with a log-rank test being used to gauge significance. Chi-squared tests were used to compare composition ratios between groups, after which a Cox proportional hazards regression model was used to identify demographic variables associated with specific prognostic outcomes (reported as hazard ratios (HRs)). The performance of the resulting predictive model was then evaluated using calibration plots and concordance index (c-index) values, with higher c-index values corresponding to superior discriminatory accuracy among possible subject outcomes (value range: 0.5-1.0). The overall agreement between predicted and observed survival outcomes was estimated via nomogram plot calibration, as in previous studies [14, 15]. We additionally employed an internal verification approach in order to predict survival outcomes in a separate conjunctival cancer patient cohort. The accuracy of these predictions was evaluated based upon the area under the receiver operating characteristic (ROC) curve. R (v3.6.1) and GraphPad Prism 7.00 were used for all statistical testing, with a two-sided *P* < 0.05 s the significance threshold.

## 3. Results

### 3.1. Baseline Patient Characteristics

By querying the SEER database, we were able to identify 2369 total conjunctival cancer patients, including 836 that had been diagnosed from 1992 to 2001 and 1533 that had been diagnosed from 2002 to 2011 (Table 1). In the 1992-2001 cohort, there were 32 (3.8%), 179 (21.4%), 276 (33.0%), and 349 (41.7%) patients in the <30-, 30-49-, 50-69-, and ≥70-year-old age groups. In the 2002-2011 cohort, there were 76 (5.0%), 276 (18.0%), 596 (38.9%), and 585 (38.2%) patients in the <30-, 30-49-, 50-69-, and ≥70-year-old age groups. In the 1992-2001 cohort, 321 (38.9%) patients were female and 515 (61.6%) were male, whereas in the 2002-2011 cohort, 905 (59.0%) patients were female and 628 (41.0%) were male. The majority of patients were Caucasian in both groups, with rates of 84.9% (710/836) and 84.5% (1295/1533) in the 1992-2001 and 2002-2011 cohorts, respectively. The most prevalent marital status among these patients was married (including common law marriage), with rates of 53.3% (446/836) and 54.1% (829/1533) in the 1992-2001 and 2002-2011 cohorts, respectively. The cause-specific death rates attributed to conjunctival cancer were 10.5% (88/836) in the 1992-2001 cohort and 6.0% (92/1533) in the 2002-2011 cohort.

### 3.2. Composition Ratio Comparisons

We next compared composition ratios between these two patient cohorts (Table 2). We observed significant differences in composition ratios corresponding to patient age groupings between the 1992-2001 and 2002-2011 cohorts (*P* = 0.009), with clear differences in the frequencies of individuals in the 30-49 and 50-69 age groups between these two groups of patients (*P* < 0.05). No significant differences in ethnicity ratios were detected between these cohorts (*P* = 0.519), but sex distributions did differ significantly between groups (*P* ≤ 0.001). With respect to marital status, there were also significant differences in the composition ratios corresponding to single and widowed status between the 1992-2001 and 2002-2011 cohorts (*P* = 0.01). Cause-specific death rate composition ratios similarly differed significantly between these two patient groups (*P* ≤ 0.001).

### 3.3. Age-Adjusted Incidence Rates

Among patients aged 50-69 years, the annual percent change (APC) in the age-adjusted incidence rate trend in patients between 1992-2001 and 2002-2011 was -1.5^∗^ (*P* < 0.05) (Table 3), indicating a significant reduction in the age-adjusted incidence rate in this cohort in the latter decade relative to the former decade. All other incidence trends in this study were found to be stable over time.

### 3.4. Cause-Specific Survival

We further determined the 1-, 3-, and 5-year cause-specific survival rates for these 1992-2001 and 2002-2011 patient cohorts (Table 4). With increasing follow-up time, the cause-specific age std and cause-specific survival rates decreased. Relative to the 1992-2001 patient cohort, these values tended to rise if the 2002-2011 patient cohort tended to increase.

### 3.5. Comparison of Overall Survival between Patient Cohorts

We observed no significant differences in overall survival (OS) between the 1992-2001 and 2002-2011 patient cohorts (*P* = 0.1290) (Figure 1).

We observed significant differences in OS rates among patients in the <30-, 30-49-, 50-69-, and ≥70-year-old age groups (Figure 2). Specifically, patients ≥ 70 years old exhibited significantly poorer OS than did patients of other ages (*P* < 0.0001), while patients aged 50-69 years exhibited relatively higher OS relative to patients aged 30-49 years (1992-2001: *P* = 0.0009; 2002-2011: *P* = 0.0010) and patients aged <30 years (*P* < 0.0001). There was a significant difference in the OS of patients < 30 years old relative to patients aged 30-49 years (*P* = 0.0056).

Survival rates also differed significantly between males and in both the 1992-2001 cohort (*P* = 0.0050) and the 2002-2011 cohort (*P* < 0.0001), with females having a better average OS than males (Figure 3).

While there was no significant difference in OS as a function of ethnicity in the 1992-2001 cohort (*P* = 0.1124), such differences were evident in the 2002-2011 cohort (*P* = 0.0021) (Figure 4). No significant differences in OS were observed in white patients relative to black patients (1992-2001: *P* = 0.9929; 2002-2011: *P* = 0.0780) while significant differences were observed for patients of other races relative to white patients (1992-2001: *P* = 0.0369; 2002-2011: *P* = 0.0018). Differences in OS were not significant when comparing patients of other races and black patients (1992-2001: *P* = 0.1650; 2002-2011: *P* = 0.3642).

There were significant differences in OS as a function of marital status in both the 1992-2001 cohort (*P* < 0.0001) and the 2002-2011 cohort (*P* < 0.0001) (Figure 5). Specifically, patients who were single exhibited significantly poorer OS than did patients that were married (*P* < 0.0001), widowed (*P* < 0.0001), or divorced (*P* = 0.0004). No significant differences in OS were observed between patients that were married and those that were widowed (*P* = 0.1130), divorced (*P* = 0.2856), or separated (*P* = 0.5907). OS values for patients that were single did not differ significantly from those of patients that were separated (*P* = 0.2128). Similarly, OS values for patients that were widowed did not differ significantly from those of patients that were divorced (*P* = 0.0686) or separated (*P* = 0.3118), and survival rates were comparable between divorced and separated patients (*P* = 0.8115). There was no significant difference in OS between single and married patients (*P* = 0.1122), but widowed patients exhibited significantly worse OS than did married patients (*P* < 0.0001).

The survival rates of married patients did not differ significantly from those of divorced (*P* = 0.5369) or separated (*P* = 0.0808) patients. The OS of divorced patients was significantly poorer than that of single patients (*P* < 0.0001). Single patient survival did not differ significantly from that of separated patients (*P* = 0.1143), nor did the survival of divorced and separated patients (*P* = 0.0615).

### 3.6. Nomogram

We next constructed a predictive nomogram incorporating survival-related variables as a means of estimating the 3- and 5-year OS of patients in this study (Figure 6). This nomogram allows for the calculation of a putative OS value for patients based on the addition of specific variables corresponding to patient demographic characteristics. This nomogram achieved a c-index value of 0.727 ((a) 1992-2001), 0.747 ((b) 2002-2011), and 0.736 ((c) 1992-2011) consistent with a relatively good discriminative ability (in Table 5).

Calibration plots assessing the predictive accuracy of this nomogram are shown in Figure 7(a) (1992-2001), 7(b) (2002-2011) and 7(c) (1992-2011). These plots confirm that there was good agreement between the predicted and actual 3- and 5-year OS values.

### 3.7. Cox Regression Model

The results of our Cox proportional hazards regression analysis are compiled in Table 5. This analysis revealed that being 50-69 years old (*P* < 0.01), ≥70 years old (*P* < 0.001), male (*P* < 0.001), single (*P* < 0.001), and divorced (*P* < 0.05) were all independently associated with survival outcomes in the 1992-2001 patient cohort (Table 5(a)). Similarly, this approach revealed that being male (*P* < 0.001) and single (*P* < 0.001) were both independently associated with survival outcomes in the 2002-2011 patient cohort (Table 5(b)). An additional regression analysis was conducted for the overall patient population in this study, revealing that being 30-49 years old (*P* < 0.05), 50-69 years old (*P* < 0.001), ≥70 years old (*P* < 0.001), of another race (*P* < 0.05), male (*P* < 0.001), single (*P* < 0.05), widowed (*P* < 0.001), or divorced (*P* < 0.001) were all independently associated with survival (Table 5(c)).

### 3.8. Nomogram Validation

We next sought to evaluate the accuracy of our nomograms as a means of predicting conjunctival cancer patient outcomes using clinical data from a large separate patient cohort. For internal validation purposes, we utilized receiver operating characteristic (ROC) curves and measured the area under the curve (AUC) (Figure 8). These analyses revealed relatively strong predictive abilities, with 3- and 5-year AUC values of 0.715 (a) and 0.74166 (b) in standard mode, respectively, and 0.697 (c) and 0.75249 (d) in verification mode, respectively.

## 4. Discussion

Overall, the results of our analysis suggest that primary site-labeled conjunctival cancer rates and outcomes have been relatively stable over the past 20 years. We detected no significant differences in OS between the 1992-2001 and 2002-2011 patient cohorts. We did, however, detect a significant decrease in the age-adjusted incidence of conjunctival cancer in the 50-69-year-old age group over this time period in 2002-2011 patient cohorts (APC; *P* < 0.05). Age is the traditional primary risk factor in many diseases, especially in cancer. At present, the age distribution of the world population tends to be aging. Growth of the older population leads to changes in the age distribution, cancer spectrum, and mortality of cancer patients. Age-adjusted statistics are recommended to better reflect the effects of age structure changes on cancer epidemiological outcomes.

We observed significant relationships between specific demographic variables and conjunctival cancer incidence. Specifically, we found that being ≥30 years of age (*P* < 0.05), male (*P* < 0.001), single (*P* < 0.05), divorced (*P* < 0.001), and widowed (*P* < 0.001) were all risk factors associated with primary conjunctival cancer incidence in the overall study cohort, whereas being of a race designated as “other” was identified as a protective factor (Table 5(c)).

The incidence of primary conjunctival and corneal malignancies has previously been shown to be associated with patient age. In our overall study cohort, there were patients of all ages with such tumors including patients < 1 year old and >100 years old. We did, however, observe an increase in the incidence of these tumors with increasing age, particularly in persons > 50 years old. Such age-related trends towards increased incidence have also been previously observed in children, with a prior study demonstrating that the mean age at detection was 11 years for nonmalignant tumors and 14 years for malignant tumors (*P* = 0.005), with a mean three-year difference in detection (95% CI, 1.2-4.6) [6]. We were able to confirm that patient age was significantly related to both primary conjunctival and corneal cancer incidence and the OS of affected individuals (Figure 2 and Table 5(c)). It is therefore important that the differential diagnosis of conjunctival and corneal cancers be considered, particularly in elderly patients, with a pathological assessment being conducted as appropriate.

We observed no significant differences in the age-corrected incidence of conjunctival and corneal cancer when comparing patient cohorts from 1992 to 2001 and 2002 to 2011, although we did detect a downward incidence trend specifically in the 50-69-year-old age group (APC = −1.5). This may be related to both the low overall incidence of these cancers, increased awareness thereof, and/or an increase in preventative measures among this population. Together, these results emphasize that the incidence of primary site-labeled conjunctival cancer over the last two decades is relatively stable. Using these data, we were also able to construct a nomogram that was shown to have relatively good predictive accuracy (Figure 7) and satisfactory AUC values (Figure 8) for both the overall patient cohort and the individual decade cohorts. These models also suggested that the prognosis of conjunctival and corneal cancers has similarly remained stable over this 20-year period. Malignant conjunctival and corneal tumors are relatively rare, with squamous cell carcinoma (SCC) being the most prevalent form of conjunctival malignancy with a 0.02-3.5 per 100,000 incidence rate. In contrast, the incidence rate of conjunctival melanoma is lower (0.24-0.53 per 1,000,000) [16]. The survival rate of conjunctival cancer is relatively high, potentially because these tumors are easy to identify, observe, and biopsy, allowing for more timely treatment and follow-up [10].

The results of our Cox regression analysis suggest that being male is associated with an elevated risk of developing malignant conjunctival tumors (Table 5). Yu et al. previously found that over the 27-year period from 1973 to 1999, the incidence of conjunctival malignancies rose by 295% in white males [17]. Another study has shown that ocular surface squamous neoplasms are more frequently detected in males, with a male-to-female ratio of 3.3 : 1.0 [18]. More recent studies have similarly observed sex-related differences in conjunctival tumor incidence in different age groups, including in pediatric patients [7]. Conjunctival lymphomas are most commonly detected in elderly individuals (60-70 years old), with extranodal marginal zone (EMZL) being more common in female patients (57.8% (104 of 180)) and mantle cell lymphoma (MCL) being predominantly detected in males (77.8% (14 of 18)) [19]. However, other analyses have suggested that sex is not associated with conjunctival or corneal tumor incidence or prognosis [20]. No specific explanation as to why men are at a higher risk of such tumors has been defined [21], but relevant risk factors could include differences in UV exposure, outdoor activity, hormones, study populations, or analyzed tumor types. Further study of the relative incidence of malignant conjunctival tumors in males and females is thus warranted.

Our study is the first to demonstrate that being single, divorced, or widowed is a risk factor associated with primary site-labeled conjunctival and corneal cancer incidence. Prior studies have primarily only examined the relationship between marital status and other forms of cancer including colorectal cancer [22], neuroendocrine tumors [23], and gastric adenocarcinoma [24] in retrospective [25] analyses or in prospective analyses [26]. While several studies have assessed the relationship between marital status and patient prognosis, conclusions have varied significantly among studies. Our results do not provide any insight into the relationship between these variables, but they do suggest that social relationships may impact patient psychological state, nursing care, follow-up, or treatment choice. Further study of this result is warranted in order to properly guide patient care in an efficacious fashion.

Malignant conjunctival tumor prognosis is related to many factors not assessed in the present study (because of the rarity of some data), including tumor type, lesion size, overall patient health, interventions used, and follow-up. For example, mucoepidermoid carcinoma is more common in older patients and is typically more aggressive than squamous cell cancer (SCC), necessitating wider excision and closer follow-up [27]. Conjunctival SCC in immunosuppressed patients can also be more invasive and aggressive than in healthy patients, requiring enucleation or exenteration. In such patients, the risk of disease-associated mortality is significantly elevated [12]. Melanomas > 1.0 mm in size are associated with mortality rates of 33-50% regardless of whether exenteration was conducted as a primary or secondary treatment, with caruncular melanomas having a particularly poor prognosis regardless of exenteration, emphasizing the importance of early-stage complete tumor removal when possible [28].

In summary, the results of this study suggest that the incidence and prognosis of primary site-labeled conjunctival cancer have remained relatively stable over the past two decades, consistent with previous reports. Even so, it is important that such tumors be diagnosed and treated in an individualized manner based upon local differences in tumor epidemiology and in light of the experience of individual clinicians.

## Figures and Tables

**Figure 1:** Conjunctival cancer overall survival rates were estimated via the Kaplan-Meier approach between the 1992-2001 and 2002-2011 patient cohorts (*P* = 0.1290).

**Figure 2:** Kaplan-Meier estimate of the overall survival of specific age groups in the 1992-2001 and 2002-2011 patient cohorts.

**Figure 3:** Kaplan-Meier estimate of overall survival as a function of sex in the 1992-2001 and 2002-2011 patient cohorts.

**Figure 4:** Kaplan-Meier estimate of overall survival as a function of ethnicity in the 1992-2001 and 2002-2011 patient cohorts.

**Figure 5:** Kaplan-Meier estimate of overall survival as a function of marital status in the 1992-2001 and 2002-2011 patient cohorts.

**Figure 6:** A nomogram including the variables independently related to survival is shown. (a) Variables independently related to survival in group 1992-2001; (b) variables independently related to survival in group 2002-2011; (c) variables independently related to survival in group 1992-2011.

**Figure 7:** Calibration plots of the nomogram predictions of 3-year and 5-year overall survival of conjunctival cancers in the (a) 1992-2001, (b) 2002-2011, and (c) 1992-2011 patients cohorts. The blue line represents equivalence between the observed and predicted probabilities.

**Figure 8:** Receiver operating characteristic (ROC) curves and measurements of the area under the curve (AUC) as a means of evaluating model accuracy. (a) 3-year AUC in standard mode. (b) 5-year AUC in standard mode. (c) 3-year AUC in verification mode. (d) 5-year AUC in verification mode.

**Table 1:** Overview of the 2369 patients in the study cohort 1992-2001/2002-2011.

Characteristic	No. (%) of patients (1992-2001)	No. (%) of patients (2002-2011)
Age		
<30	32 (3.8%)	76 (5.0%)
30-49	179 (21.4%)	276 (18.0%)
50-69	276 (33.0%)	596 (38.9%)
≥70	349 (41.7%)	585 (38.2%)
Status		
Alive	346 (41.4%)	984 (64.3%)
Dead	490 (58.6%)	549 (35.8%)
Race		
White	710 (84.9%)	1295 (84.5%)
Other (American Indian/AK Native, Asian/Pacific Islander)	70 (8.4%)	108 (7.0%)
Black	40 (4.8%)	79 (5.2%)
Unknown	16 (1.9%)	51 (3.3%)
Sex		
Female	321 (38.4%)	905 (59.0%)
Male	515 (61.6%)	628 (41.0%)
Specific_death_Cause		
Alive or dead of other cause	624 (74.6%)	1133 (73.9%)
Dead (attributable to this cancer dx)	88 (10.5%)	92 (6.0%)
Dead (missing/unknown COD)	9 (1.1%)	8 (0.5%)
N/A not first tumor	115 (13.8%)	300 (19.6%)
Marital_status		
Divorced	52 (6.2%)	80 (5.2%)
Married (including common law)	446 (53.3%)	829 (54.1%)
Separated	3 (0.4%)	7 (0.5%)
Single (never married)	104 (12.4%)	232 (15.1%)
Unknown	109 (13.0%)	231 (15.1%)

**Table 2:** Composition ratios between 1992-2001 and 2002-2011.

Characteristic	1992-2001	2002-2011	*P*
Age			
<30	32^a^	76^a^	*P* = 0.009
30-49	179^a^	276^b^	
50-69	276^a^	596^b^	
≥70	349^a^	585^a^	
Race			
White	710^a^	1295^a^	*P* = 0.519
Other (American Indian/AK Native, Asian/Pacific Islander)	70^a^	108^a^	
Black	40^a^	79^a^	
Sex			
Female	321^a^	905^b^	*P* ≤ 0.001
Male	515^a^	628^b^	
Specific_death_Cause			
Alive or dead of other cause	624^a^	1133^b^	*P* ≤ 0.001
Dead (attributable to this cancer dx)	88^a^	92^b^	
Marital_status			
Divorced	52^a^	80^a^	*P* = 0.01
Married (including common law)	446^a^	829^a^	
Separated	3^a^	7^a^	
Single (never married)	104^a^	232^b^	
Widowed	122^a^	154^b^	

a, a: means *P* > 0.05 between group 1992-2001 and group 2002-2011. a, b: means *P* < 0.05 between group 1992-2001 and group 2002-2011.

**Table 3:** Incidence rate trends (age-adjusted).

Characteristic	APC
Sex	
Female and male	-0.4
Female	-1.7
Male	0.3
Race	
All races	-0.1
White	0.0
Black	
Other (American Indian/AK Native, Asian/Pacific Islander)	-2.3
Age	
All ages	-0.4
<30	-5.8
30-49	-2.8
50-69	-1.5^∗^
≥70	1.6

∗: the APC differed significantly from that for 1992-2001 (*P* < 0.05).

**Table 4:** Cause-specific survival.

Group	Time	Cause-specific age Std	Cause-specific	SE cause-specific age Std	SE cause-specific
1992-2001	1 y	96.60%	96.50%	0.90%	0.90%
	3 y	87.00%	87.70%	1.80%	1.60%
	5 y	76.30%	78.60%	2.20%	2.10%
2002-2011	1 y	95.40%	95.70%	1.20%	1.00%
	3 y	91.00%	91.40%	1.60%	1.50%
	5 y	83.00%	84.80%	2.40%	2.10%

Abbreviations: SE: standard error; Std: standard deviation.

**Table:** (a) 1992-2001 Cox proportional hazards regression

Concordance = 0.727 (SE = 0.012)				
	coef	exp(coef)	SE(coef)	*P*
Age 30-49	5.906*E* − 01	1.805*E* + 00	6.132*E* − 01	3.355*E* − 01
Age 50-69	1.750*E* + 00	5.753*E* + 00	5.970*E* − 01	3.380*E* − 03^∗∗^
Age ≥ 70	2.944*E* + 00	1.898*E* + 01	5.949*E* − 01	7.520*E* − 07^∗∗∗^
Race black	2.134*E* − 01	1.238*E* + 00	2.258*E* − 01	3.447*E* − 01
Race other	−1.794*E* − 01	8.358*E* − 01	1.974*E* − 01	3.633*E* − 01
Sex male	5.536*E* − 01	1.740*E* + 00	1.116*E* − 01	7.020*E* − 07^∗∗∗^
marital_Single	5.183*E* − 01	1.679*E* + 00	1.309*E* − 01	7.480*E* − 05^∗∗∗^
marital_Widowed	2.785*E* − 01	1.321*E* + 00	1.677*E* − 01	9.671*E* − 02
marital_Divorced	4.248*E* − 01	1.529*E* + 00	1.947*E* − 01	2.915*E* − 02^∗^
marital_Separated	5.470*E* − 02	1.056*E* + 00	5.838*E* − 01	9.252*E* − 01

**Table:** (b) 2002-2011 Cox proportional hazards regression

Concordance = 0.747 (SE = 0.011)				
	coef	exp(coef)	SE(coef)	*P*
Age 30-49	1.639*E* + 01	1.307*E* + 07	1.206*E* + 03	9.892*E* − 01
Age 50-69	1.702*E* + 01	2.455*E* + 07	1.206*E* + 03	9.887*E* − 01
Age ≥ 70	1.831*E* + 01	8.987*E* + 07	1.206*E* + 03	9.879*E* − 01
Race black	1.417*E* − 01	1.152*E* + 00	2.316*E* − 03	5.407*E* − 01
Race other	−4.080*E* − 01	6.650*E* − 01	2.355*E* − 01	8.320*E* − 02
Sex male	5.111*E* − 01	1.667*E* + 00	1.024*E* − 01	6.020*E* − 07^∗∗∗^
marital_Single	2.784*E* − 01	1.321*E* + 00	1.450*E* − 01	5.490*E* − 02^∗∗∗^
marital_Widowed	7.223*E* − 01	2.059*E* + 00	1.240*E* − 01	5.650*E* − 09
marital_Divorced	3.321*E* − 01	1.394*E* + 00	1.965*E* − 01	9.100*E* − 02
marital_Separated	−1.671*E* + 01	5.541*E* − 08	3.180*E* + 03	9.958*E* − 01

**Table:** (c) 1992-2011 Cox proportional hazards regression

Concordance = 0.736 (SE = 0.008)				
	coef	exp(coef)	SE(coef)	*P*
Age 30-49	1.228*E* + 00	3.415*E* + 00	5.204*E* − 01	1.826*E* − 02^∗^
Age 50-69	2.149*E* + 00	8.574*E* + 00	5.096*E* − 01	2.480*E* − 05^∗∗∗^
Age ≥ 70	3.398*E* + 00	2.989*E* + 01	5.081*E* − 01	2.280*E* − 11^∗∗∗^
Race black	1.460*E* − 01	1.157*E* + 00	1.612*E* − 01	3.649*E* − 01
Race other	−3.015*E* − 01	7.397*E* − 01	1.506*E* − 01	4.528*E* − 02^∗^
Sex male	5.443*E* − 01	1.723*E* + 00	7.509*E* − 02	4.180*E* − 13^∗∗∗^
marital_Single	2.739*E* − 01	1.315*E* + 00	1.095*E* − 01	1.238*E* − 02^∗^
marital_Widowed	6.252*E* − 01	1.869*E* + 00	8.962*E* − 02	3.020*E* − 12^∗∗∗^
marital_Divorced	3.662*E* − 01	1.442*E* + 00	1.377*E* − 01	7.840*E* − 03^∗∗∗^
marital_Separated	−4.329*E* − 01	6.486*E* − 01	5.807*E* − 01	4.560*E* − 01

Abbreviations: SE: standard error. coef: coefficient. *P*: *P* value. ∗: *P* < 0.05, ∗∗: *P* < 0.01, ∗∗∗: *P* < 0.001.

## Data Availability

The datasets generated and analyzed being used for this study are available from the Surveillance, Epidemiology, and End Results (SEER) database from 1992 to 2001 and from 2002 to 2011. SEER∗Stat 8.3.6 is available on https://seer.cancer.gov/.
